The article "Physiological and biochemical responses of Kinnow mandarin grafted on diploid and tetraploid Volkamer lemon rootstocks under different water-deficit regimes" was retracted in 2022. Reasons: compromised peer review; a conflict of interest; concerns about the authorship.

# Physiological and biochemical responses of Kinnow mandarin grafted on diploid and tetraploid Volkamer lemon rootstocks under different water-deficit regimes

**DOI:** 10.1371/journal.pone.0247558

**Published:** 2021-04-08

**Authors:** Muhammad Fasih Khalid, Sajjad Hussain, Muhammad Akbar Anjum, Raphael Morillon, Shakeel Ahmad, Shaghef Ejaz, Mubshar Hussain, Hawa Z. E. Jaafar, Sara T. Alrashood, Alexe Nicolae Ormenisan

**Affiliations:** 1 Faculty of Agricultural Sciences and Technology, Department of Horticulture, Bahauddin Zakariya University, Multan, Pakistan; 2 Equipe “Structure Evolutive des Agrumes, Polyploidie et Amelioration Genetique, SEAPAG- CIRAD, UMR AGAP, Petit-Bourg, Guadeloupe, France; 3 AGAP, Univ Montpellier, CIRAD, INRAE, Institut Agro, Montpellier, France; 4 Faculty of Agricultural Sciences and Technology, Department of Agronomy, Bahauddin Zakariya University, Multan, Pakistan; 5 Faculty of Agriculture, Department of Crop Science, University Putra Malaysia, UPM Serdang, Selangor, Malaysia; 6 Department of Pharmaceutical Chemistry, College of Pharmacy, King Saud University, Riyadh, Saudi Arabia; 7 Department of Food and Tourism Engineering and Management, Transilvania University of Brasov, Brasov, Romania; Harran Üniversitesi: Harran Universitesi, TURKEY

## Abstract

Water shortage is among the major abiotic stresses that restrict growth and productivity of citrus. The existing literature indicates that tetraploid rootstocks had better water-deficit tolerance than corresponding diploids. However, the associated tolerance mechanisms such as antioxidant defence and nutrient uptake are less explored. Therefore, we evaluated physiological and biochemical responses (antioxidant defence, osmotic adjustments and nutrient uptake) of diploid (2x) and tetraploid (4x) volkamer lemon (VM) rootstocks grafted with kinnow mandarin (KM) under two water-deficit regimes. The KM/4xVM (VM4) and KM/2xVM (VM2) observed decrease in photosynthetic variables, i.e., photosynthetic rate (*Pn*), stomatal conductance (*g*_*s*_), transpiration rate (*E*), leaf greenness (SPAD), dark adopted chlorophyll fluorescence (Fv/Fm), dark adopted chlorophyll fluorescence (Fv´/Fm´), relative water contents (RWC) and leaf surface area (LSA), and increase in non-photochemical quenching (NPQ) under both water-deficit regimes. Moreover, oxidative stress indicators, i.e., malondialdehyde (MDA) and hydrogen peroxide, and activities of antioxidant enzymes, i.e., superoxide dismutase (SOD), peroxidase (POD), catalase (CAT), ascorbate peroxidase (APx), glutathione reductase (GR) were increased under both water-deficit regimes. Nonetheless, increase was noted in osmoprotectants such as proline (PRO) and glycine betaine (GB) and other biochemical compounds, including antioxidant capacity (AC), total phenolic content (TPC) and total soluble protein (TSP) in VM2 and VM4 under both water-deficit regimes. Dry biomass (DB) of both rootstocks was decreased under each water-deficit condition. Interestingly, VM4 showed higher and significant increase in antioxidant enzymes, osmoprotectants and other biochemical compounds, while VM2 exhibited higher values for oxidative stress indicators. Overall, results indicated that VM4 better tolerated water-deficit stress by maintaining photosynthetic variables associated with strong antioxidant defence machinery as compared to VM2. However, nutrient uptake was not differed among tested water-deficit conditions and rootstocks. The results conclude that VM4 can better tolerate water-deficit than VM2. Therefore, VM4 can be used as rootstock in areas of high-water deficiency for better citrus productivity.

The article "Physiological and biochemical responses of Kinnow mandarin grafted on diploid and tetraploid Volkamer lemon rootstocks under different water-deficit regimes" was retracted in 2022. Reasons: compromised peer review; a conflict of interest; concerns about the authorship.

## Introduction

Citrus plays a vital role in economy of many developed and developing countries. However, citrus greening disease (Huanglongbing) is decreasing citrus productivity, which ultimately affects fruit and juice prices [1]. Numerous other factors such as abiotic stresses also decrease citrus production. Drought is probably the most important among abiotic stresses decreasing citrus productivity. Citrus trees require short-term water deficiency for flowering induction; however, long-term water deficiency negatively affects plant growth and yield [2,3]. Water deficiency causes stomatal closure, which decreases the efficiency of photosynthetic machinery and limits transportation of water and solutes to tree canopy [4]. Plants restricts water loss under water stress by hardening cell wall and undergo some metabolic changes, i.e., production of proteins and osmolytes etc. [5]. Production of different reactive oxygen species (ROS) is also increased under stressed conditions. These ROS may alter the metabolic process in mitochondria and chloroplast [6]. Plant defence machinery produces different scavenging enzymes and osmoprotectants to overcome the production of ROS [7,8]. Citrus rootstocks can behave differently depending on the defence mechanism against water-deficit condition [8]. Drought tolerant rootstocks have higher capability to maintain their photosynthetic mechanism through strong defence machinery [8–10]. Citrus are diploid (2x), but spontaneous polyploid citrus rootstocks are produced through mitotic division of somatic embryos [11]. Tetraploid (4x) (4n = 36) rootstocks have different traits than their 2x parent. Tetraploid citrus seedlings are known to have higher tolerance to different abiotic stresses than 2x seedlings [9,12–14]. Nonetheless, similar findings have been reported for grafted tress under water-deficit conditions [11]. Diploid root stocks have thinner leaves and less chlorophyll content than 4x. Tetraploid rootstocks have shorter and thicker roots, which results in slower growth [15,16]. All these anatomical and physiological changes do not affect fruit quality of scions grafted on 4x rootstock [17]. Rootstock-scion combination affects growth, yield and induces tolerance against different biotic and abiotic stresses [18]. However, if rootstock-scion relationship is not successful, it may cause barriers in water and mineral nutrients translocation resulting in callus formation and altered physiological and biochemical processes [19]. Climate change is resulting in two types of water-deficit stress, which negatively affect citrus production. These include short and severe stress, and slow and prolonged stress. It is expected that plants would show quick response by closing stomata under fast water-deficit stress. However, plants will have more time to adapt to slow and prolonged water-deficit and slowly close the stomata. Nonetheless, ROS scavenging response under both type of stresses is still elusive. Few studies have inferred the response of citrus to both types of stresses; however, none of these analysed the defence machinery of kinnow mandarin grafted on 2x and 4x rootstocks.

The article "Physiological and biochemical responses of Kinnow mandarin grafted on diploid and tetraploid Volkamer lemon rootstocks under different water-deficit regimes" was retracted in 2022. Reasons: compromised peer review; a conflict of interest; concerns about the authorship.

Therefore, we investigated the impact of quick and slow water-deficit stress on the physiological and biochemical responses of 2x and 4x Volkamer lemon (*Citrus volkameriana* Tan. and Pasq) rootstocks grafted with Kinnow mandarin (*Citrus nobilis* x *Citrus deliciosa*). It was hypothesized that both rootstocks will show differential response to both stresses and 4x would had better drought tolerance. The results of the study will help to identify the tolerance mechanisms and select the best-suited rootstock for drought-prone areas.

## Materials and methods

### Plant material

Diploid (2x) and tetraploid (4x) Volkamer lemon (*Citrus volkameriana* Tan. and Pasq.) seeds were obtained from Centre of International Research on Agriculture and Development (CIRAD), France. Seeds were sown in plastic container for 3 months. Afterwards, homogenous plants were selected and the zygotic and nucellar status of seedlings was confirmed by using 13 SSR markers advised by Luro et al. [20]. The 2x and 4x ploidy level of selected rootstocks were checked by flow cytometry [21]. After six months, similar and healthy plants from each rootstock were selected and grafted with Kinnow mandarin (*Citrus nobilis* × *Citrus deliciosa*). Plants were exposed to water-deficit treatments one year after grafting. The plants were placed in 30 cm pot filled with sandy-loam soil. Plants were divided in two groups and placed in greenhouse under 28 °C day and 18 °C night temperature along with 50 to 70% relative humidity. Each group had control (well-watered) and treated (water-deficit) pots. In water-deficit condition, we completely stopped irrigation after attaining maximum water holding capacity of pots. Water-deficit conditions consisted of fast and strong lowering of the soil water potential, and slow and limited lowering of the soil water potential. The slow and limited lowering water-deficit was attained by covering the top of the pots, which slowed transpiration stream. Plants were regularly irrigated to field capacity for 2 weeks before initiating water-deficit treatments. The experiment was conducted in randomized complete block design with three replicates. Four plants were placed in each replication (two for destructive samplings and two for non-destructive sampling). The water-deficit treatments prevailed for 9 days and data relating to physiological and biochemical attributes were recorded at the termination of water-deficit treatments.

The article "Physiological and biochemical responses of Kinnow mandarin grafted on diploid and tetraploid Volkamer lemon rootstocks under different water-deficit regimes" was retracted in 2022. Reasons: compromised peer review; a conflict of interest; concerns about the authorship.

### Attributes studied

Two leaves per plant were randomly selected to measure photosynthetic variables. In case of leaf senescence, the adjacent leaves were used. Leaves were measured every 3 days for the measurement of biometric variables. Antioxidant enzymes, osmolytes and nutrient uptake in leaves and roots were measured at the end of the experiment. Root dry weight was measured taking off the plants from the pots. All samplings and measurements were carried out between 9 AM– 11 AM.

### Photosynthetic variables

Leaf photosynthetic variables, photosynthetic rate (*Pn*), transpiration rate (*E*) and stomatal conductance (*g*_*s*_) were measured with infrared gas analyser (ADC, BioScientific Ltd. UK). Indirect measurement of chlorophyll was made with the help of SPAD meter (Konica Minolata SPAD-502. Japan). Chlorophyll fluorescence in light-acclimated (Fv´/Fm´), dark-acclimated (Fv/Fm) leaves and non-photochemical quenching (NPQ) in dark-acclimated leaves were measured with a chlorophyll fluorometer (FluorPen FP-100. Czech Republic).

Fresh weight of leaves was taken by a weighing balance, afterwards leaves were soaked in water for 12 hours for saturation and weighed. The leaves were then dried in oven at 62 °C for 72 hours to measure the relative water content (RWC) as advised by Hussain et al. [8]. Leaf surface area (LSA) was measured by laser leaf area meter (CI-202, CID, USA).

Leaves and roots samples from destructive sampling plants were harvested and crushed in liquid nitrogen to stop the activity. Crushed samples were used for determination of enzymatic activities, osmolytes and other biochemical parameters.

The article "Physiological and biochemical responses of Kinnow mandarin grafted on diploid and tetraploid Volkamer lemon rootstocks under different water-deficit regimes" was retracted in 2022. Reasons: compromised peer review; a conflict of interest; concerns about the authorship.

### Activities of antioxidant enzymes

For the estimation of superoxide dismutase (SOD), catalase (CAT) and peroxidase (POD) activities, 0.3 gram leaf and root samples were taken in chilled mortar and pestle, and homogenized with 50 mM sodium phosphate buffer (7.8 pH).

For SOD activity methods of Giannopolitis and Ries [22] were followed. The solution was formulated with 75 mM ethylenediaminetetraacetic acid, 50 μM nitroblue tetrazolium, 50 mM sodium phosphate buffer (pH 7.8), 1.3 μM riboflavin, 13 mM methionine and enzyme extract were added and absorbance was checked at 560 nm wavelength through UV-1900 spectrophotometer (BMS, Canada). The CAT activity was measured by the method of Chance and Maehly [23]. The mixture contained 5.9 mM hydrogen peroxide, 50 mM sodium phosphate buffer (7.8 pH) and extracted enzyme. The absorbance at 240 nm wavelength was measured by UV-1900 spectrophotometer (BMS, Canada). The POD activity was estimated by the method of Chance and Maehly [23]. Mixture contained 20 mM guaiacol, 50 mM sodium phosphate buffer (7.8 pH), 40 mM hydrogen peroxide and enzyme extract. The absorbance for POD were noted at 470 nm wavelength.

Ascorbate peroxidase (APx) activity was measured as advised by Nakano and Asada [24]. The solution contained 50 mM sodium phosphate buffer (7.0 pH), 0.5 mM ascorbate, 0.1 mM ethylenediaminetetraacetic acid, 1.2 mM hydrogen peroxide and enzyme extract. The absorbance was read at wavelength of 290 nm. For estimation of glutathione reductase (GR) activity, method of Foyer and Halliwell [25] was followed. Solution contained 100 mM potassium phosphate buffer (7.8 pH), 0.5 mM glutathione oxidised form, 0.2 mM nicotinamide adenine dinucleotide phosphate, 2 mM ethylenediaminetetraacetic acid and extracted enzyme. The absorbance of the solution was noted at 340 nm by spectrophotometer.

### Determination of osmoprotectants

For the determination of proline, 0.5 g freshly harvested leaves and roots were homogenized in 3% sulfosalicylic acid as advised by Bates et al. [26]. The reaction solution contained ninhydrin reagent, glacial acetic acid and extracted sample. The solution was heated at 100 °C for 60 minutes in hot water bath and immediately cooled in chilled water to stop the reaction. After cooling, 4 mL toluene was added and the absorbance of supernatant was noted at 520 nm.

For glycine betaine content, estimation was done by the method of Grieve and Grattan [27]. The 0.5 g plant sample was homogenized in distilled water. The solution contained hydrochloric acid, potassium tri-iodide and extracted sample. This solution was placed in ice bath for 90 minutes and continuously shaken. Then chilled distilled water and chilled 1, 2-dichloroethane was added in the solution. Lower layer was used and its absorbance was noted at 365 nm.

The article "Physiological and biochemical responses of Kinnow mandarin grafted on diploid and tetraploid Volkamer lemon rootstocks under different water-deficit regimes" was retracted in 2022. Reasons: compromised peer review; a conflict of interest; concerns about the authorship.

### Hydrogen peroxide, malondialdehyde and total soluble proteins

For estimation of hydrogen peroxide and malondialdehyde, 0.2 g freshly harvested leaves and roots were homogenized in 0.1% trichloroacetic acid.

Hydrogen peroxide was estimated by the method of Velikova et al. [28]. The reaction solution contained 1 M potassium iodide, 10 mM potassium phosphate buffer and extracted sample. The absorbance of solution was noted at 390 nm through spectrophotometer. Malondialdehyde (MDA) was measured as described by Heath and Packer [29]. The solution contained 0.5% thiobarbituric acid, 20% trichloroacetic acid and extracted sample. The solution was heated at 100 °C and immediately cooled. The readings were estimated at 532 and 600 nm wavelength through spectrophotometer.

For estimation of total soluble proteins, 0.5 g leaf and root samples were homogenized in phosphate buffer saline (7.2 pH) according to Sambrook and Russell [30]. The reaction solution contained deionized water, coomassie blue dye and extracted plant material. The absorbance of the reaction solution was read at 595 nm wavelength.

### Antioxidant capacity and total phenolic contents

The antioxidant capacity (AC) and total phenolic content (TPC) were estimated as suggested by Ozgen et al. [31]. The 0.5 g sample of leaves and roots were homogenized in solution (70% ethanol, 29% distilled water and 1% acetic acid). For estimation of AC, solution contained 0.1 mM 2,2-diphenyl-1-picrylhydrazyl and extracted sample. The solution was placed in dark for 10 min. The absorbance was noted at 515 nm wavelength. TPC was measured by making a solution with Folin Ciocalteu’s reagent, distilled water, 7% sodium carbonate and extracted sample. The solution was placed for 120 minutes at room temperature. The absorbance was noted at 750 nm wavelength.

### Plant nutrients

Different nutrients were analyzed at the end of the experiment in leaves and roots of 2x and 4x plants. Harvested samples were oven dried for 2 days at 70 °C. Wet digestion was carried out for calcium, phosphorous, sodium, nitrogen and potassium, while dry digestion analyses was done for chloride determination. For wet digestion, 0.1 g dry samples were digested in sulfuric acid at 300 °C for 1 hour and hydrogen peroxide was added to stabilize the reaction. The nitrogen was measured by the method of Martin et al. [32]. Phosphorous was estimated by malachite green method as advised by Ohno and Zibilske [33]. Sodium, calcium and potassium were measured by flame photometer (PFP7, Jenway UK) by following the method of Ryan et al. [34]. For dry digestion, 0.1 g sample was ashed in muffle furnace at 400 °C for 1 hour. The digested samples were homogenized in nitric acid and chloride analysis were carried out by using chloride electrode (Thermo fisher scientific, Orion 9617BNWP) and chloride standards has been made for further calculations as suggested by Hussain et al. [35].

The article "Physiological and biochemical responses of Kinnow mandarin grafted on diploid and tetraploid Volkamer lemon rootstocks under different water-deficit regimes" was retracted in 2022. Reasons: compromised peer review; a conflict of interest; concerns about the authorship.

### Statistical analysis

The data were statistically analyzed on Statistix 8.1 software. Two-way analysis of variance (ANOVA) was performed and results are summarized S2 Table. For mean comparisons, least significant difference (LSD) test at P<0.05 was used as post-hoc test. Graphs were drawn in SigmaPlot software. Principal component analysis (PCA) was performed in leaves and roots separately by RStudio.

## Results

### Gas exchange and chlorophyll fluorescence

Water loss was faster and higher in fast water-deficit treatment. Water use was higher in VM2 compared to VM4 under fast water-deficit condition (Fig 1 and S1 Table). The leaves of both rootstocks observed decrease in *Pn*, *gs*, *E* and SPAD under fast and slow water-deficit compared to control treatment. The decrease was stronger in VM2 than VM4 under both water-deficits (Fig 1). As expected, fast water-deficit had stronger impact on physiological parameters. The plants showed decrease in gas exchange attributes on 3^rd^ day of experiment under fast water-deficit, while decrease was observed at 6^th^ day under slow water-deficit (Fig 1).

**Fig 1:** Photosynthetic variables of different rootstock-scion combinations under different water-deficit regimes. (A) pot water loss; (B) photosynthesis; (C) stomatal conductance; (D) transpiration rate; (E) SPAD; (F) NPQ; (G) Fv´/Fm´; (H) Fv/Fm in the leaves of VM4 and VM2 under fast and slow water-deficit conditions. Values are mean ± S.E. at p < 0.05 (n = 3). ⚫ = VM4 control; ○ = VM2 control; ⬛ = VM4 slow water-deficit; ⬜ = VM2 slow water-deficit; ▼ = VM4 fast water-deficit; Δ = VM2 fast water-deficit.

The stress induced a decrease in Fv/Fm and Fv´/Fm´ of both rootstock-scion associations. The decrease was faster and stronger in VM2 (Fig 1). Moreover, NPQ increased under fast and slow water-deficit conditions, with higher increase noted for VM2. The change in Fv/Fm, Fv´/Fm´ and NPQ was observed on 3^rd^ day after treatment under fast and 6^th^ day in slow water-deficit (Fig 1).

### Leaf morphological responses

Both rootstocks observed a decline in RWC and LSA under both water deficits. The decrease was stronger in VM2 as compared to VM4. The decrease in RWC and LSA was faster under fast water-deficit. The decrease was recorded at 3^rd^ and 6^th^ day after the initiation of fast and slow water-deficit treatments, respectively (S1 Fig).

The article "Physiological and biochemical responses of Kinnow mandarin grafted on diploid and tetraploid Volkamer lemon rootstocks under different water-deficit regimes" was retracted in 2022. Reasons: compromised peer review; a conflict of interest; concerns about the authorship.

### Antioxidant enzyme activities and osmoprotectants

Leaves and roots of VM4 and VM2 showed increase in antioxidant enzymes activities and osmoprotectants (Figs 2 and 3). The leaves of VM4 and VM2 showed increase in the activities of SOD, CAT, APx and GR, and contents of PRO and GB. The increase was higher in VM4 as compared to VM2. The PRO content was higher in the leaves of VM2 as compared to VM4. The activity of POD increased; however, no differences were recorded between both rootstock-scion combinations (Fig 2). The activities of SOD, POD, CAT, APx and GR, and PRO and GB content in roots also increased under both water-deficit conditions. The increase was higher in VM4 than VM2 (Fig 3).

**Fig 2:** Antioxidant enzymes’ activities and osmoprotectants in the leaves of VM4 and VM2 grown under fast and slow water-deficit conditions. (A) superoxide dismutase; (B) peroxidase; (C) catalase; (D) ascorbate peroxidase; (E) glutathione reductase; (F) proline; (G) glycine betaine; (H) Total soluble proteins. ⬛ = VM4; ⬜ = VM2. Values are mean ± S.E. at p < 0.05 (n = 3).

**Fig 3:** Antioxidant enzymes’ activities and osmoprotectants in the roots of VM4 and VM2 grown under fast and slow water-deficit conditions. (A) superoxide dismutase; (B) peroxidase; (C) catalase; (D) ascorbate peroxidase; (E) glutathione reductase; (F) proline; (G) glycine betaine; (H) Total soluble proteins. ⬛ = VM4; ⬜ = VM2. Values are mean ± S.E. at p < 0.05 (n = 3).

### Hydrogen peroxide and MDA

Leaves and roots of both rootstock-scion associations recorded an increase in hydrogen peroxide and MDA contents under both water-deficit conditions (S2 and S3 Figs). The increase of hydrogen peroxide and MDA contents in leaves and roots was stronger in VM2 than VM4. Moreover, hydrogen peroxide and MDA contents were higher under fast water-deficit.

### Total soluble proteins, antioxidant capacity, total phenolic contents and dry biomass

The TSP, AC and TPC were higher in the leaves and roots of VM4 than VM2 under both water-deficits. Moreover, higher AC and TPC were recorded under fast water-deficit than slow water-deficit condition (S2 and S3 Figs). Dry biomass of leaves and roots were decreased under both water-deficits. The higher decrease was observed under fast water deficit and VM2. On the VM4 under slow water-deficit compared to control (S1 Table), while roots of VM2 showed decrease in DB under both water-deficit conditions.

### Plant nutrients

Calcium contents were increased in the leaves of both rootstock-scion combinations under stressed conditions. The increase was higher in VM2 than VM4 (Fig 4). However, calcium was increased only in the roots of VM2 under water deficit condition (Fig 5). The potassium content was decreased in the leaves of VM2 and roots of VM4 under both water-deficit regimes. Fast water-deficit resulted in a stronger decrease in potassium content as compared to slow water-deficit. The sodium content increased in the leaves of both rootstocks under both water-deficit regimes (Fig 4). The roots of VM2 recorded no change in sodium content under water deficit condition (Fig 5). Leaf chloride content did not change under tested rootstock-scion associations and water-deficit regimes (Fig 4), while a significant increase in root chloride content was observed for VM4 under slow stress (Fig 5). Nitrogen and phosphorous contents were decreased in the leaves and roots of tested rootstock-scion combinations when exposed to water deficit environment. Decrease was higher in the leaves of VM2 and roots of VM4 (Figs 4 and 5).

The article "Physiological and biochemical responses of Kinnow mandarin grafted on diploid and tetraploid Volkamer lemon rootstocks under different water-deficit regimes" was retracted in 2022. Reasons: compromised peer review; a conflict of interest; concerns about the authorship.

**Fig 4:** Nutrient accumulation in the leaves of VM4 and VM2 grown under fast and slow water deficit regimes. (A) calcium; (B) potassium; (C) sodium; (D) chloride; (E) nitrogen; (F) phosphorous. ⬛ = VM4; ⬜ = VM2. Values are mean ± S.E. at p < 0.05 (n = 3).

**Fig 5:** Nutrient accumulation in the roots of VM4 and VM2 grown under fast and slow water deficit regimes. (A) calcium; (B) potassium; (C) sodium; (D) chloride; (E) nitrogen; (F) phosphorous. ⬛ = VM4; ⬜ = VM2. Values are mean ± S.E. at p < 0.05 (n = 3).

### Multivariate analysis of leaf traits

A PCA for physiological and biochemical parameters data collected from leaves was carried out for tested rootstock-scion combinations and water-deficit regimes. The PCA separated rootstock-scion combinations under different water-deficit condition. The PC1 separated control from water deficit, whereas PC2 separated the rootstock-scion associations with different ploidy of the rootstock except for VM2. The PC1 explained 83.8% of variability in the data, while PC2 explained 5.8% variability (Fig 6).

**Fig 6:** Biplot of the first two principal components of principal component analysis executed on leaf traits of VM4 and VM2 grown under fast and slow water-deficit regimes.

### Multivariate analysis of root traits

The PCA of root traits clearly separated rootstock-scion combinations under different water-deficit condition. The PC1 separated control and deficit, whereas PC2 separated rootstock-scion combinations. A variation of 68.9% was explained by PC1 and 21% by PC2 (Fig 7).

**Fig 7:** Biplot of the first two principal components of principal component analysis executed on root traits of VM4 and VM2 grown under fast and slow water-deficit regimes.

The article "Physiological and biochemical responses of Kinnow mandarin grafted on diploid and tetraploid Volkamer lemon rootstocks under different water-deficit regimes" was retracted in 2022. Reasons: compromised peer review; a conflict of interest; concerns about the authorship.

## Discussion

Water stress restricts plant growth and development, and decreases yield of crop plants [36,37]. Pervious experiments showed that 4x citrus rootstock as seedlings and grafted with scion showed better tolerated unfavorable environmental conditions compared to their corresponding 2x [9,13,14,38]. The soil water potential were obviously different under both water-deficit regimes in the current study since water loss during the experiments was different (S1 Fig). The VM2 plants showed a higher decrease in photosynthetic attributes under fast and slow water-deficit conditions as compared to VM4 (Figs 1 and 2). When plants were exposed to water deficit conditions, *Pn* is restricted. This decrease is caused by lowered diffusion of carbon dioxide as a result of stomatal closure [39]. Moreover, tolerant citrus genotypes showed more stability in photosynthetic variables under stress conditions as compared to sensitive genotypes [9,40]. In 4x citrus plants, root to shoot signaling is mediated by several genes, i.e., *CsNCED1* which were not expressed in 2x under water deficit condition. These genes led to increases signaling to ABA from root to shoot by which plant regulate the gas exchange and resist against water deficit condition [11]. The VM4 and VM2 observed decrease in Fv/Fm and Fv´/Fm´ under water-deficit conditions. The decrease in Fv/Fm and Fv´/Fm´ was due to photo inhibitory damage and reduction in photosynthetic electron flow signaling, which is caused by photon flux density under stress conditions [41]. The NPQ increase under stress conditions was due to dissipation of damaging excess energy [2,38]. As expected, tolerant rootstock showed less decrease in Fv/Fm and Fv´/Fm´ and less increase in NPQ as compared to sensitive one [38,42]. The RWC is an important indicator of oxidative stress which decreases under water deficit condition [43,44]. The decrease in RWC is correlated with plant injury caused by the reduction in *E* [10]. A plant presenting a stronger decrease in RWC is more affected by stress [10]. The VM4 showed less decrease in RWC as compared to VM2 (Fig 3). Moreover, VM2 showed more pot water loss (Fig 2), which concluded that VM2 have higher conductivity than VM4. The VM2 showed highest decrease in plant dry biomass. Opazo et al. [45] observed that tolerant genotype showed less decrease in plant biomass as compared to sensitive genotype. As expected, higher decrease in sensitive genotype was associated with strong and early decrease in photosynthetic variables. However, root biomass of both rootstocks decreased under fast water-deficit, while under slow water-deficit root biomass of VM4 was not significantly decreased because of better water use efficiency. Therefore, there was no possibility for the trees to pool up water from deep ground, and the soil water potential was lower in VM2 than VM4 under fast water-deficit.

The article "Physiological and biochemical responses of Kinnow mandarin grafted on diploid and tetraploid Volkamer lemon rootstocks under different water-deficit regimes" was retracted in 2022. Reasons: compromised peer review; a conflict of interest; concerns about the authorship.

Lipid peroxidation indicates the cellular damage in cell membrane [46]. The MDA is the end-product of lipid peroxidation, which reacts with thiobarbituric acid [47]. When plants are subjected to water-deficit, they increase the production of ROS, which recompense the cell membrane [48]. Plants with better tolerance against water-deficit should contain less MDA and hydrogen peroxide than sensitive plants [8,38]. In our study, leaves and roots of VM2 had higher MDA and hydrogen peroxide than VM4 (S2 and S3 Figs), which is in agreement with previous work investigating tetraploid rootstocks [40].

Plant produces different scavenging enzymes, i.e., SOD, POD, CAT, APx and GR to overcome the negative effects of ROS [49]. The SOD and GR act as a catalyst. The SOD act in conversion of superoxide anion to hydrogen peroxide, while GR causes reduction in NADPH-dependent oxidized glutathione under water-deficit [8,10]. The conversion of superoxide anion ultimately decrease the production of MDA [50]. The CAT and APx detoxify hydrogen peroxide [51], while POD act as scavenging enzyme against hydrogen peroxide in chloroplast [52]. Moreover, plants also produced different osmoprotectants, i.e., PRO and GB to cope with ROS. Osmoprotectants cause reduction in ROS, helps the plant by osmotic adjustments and maintain photosynthetic machinery under unfavorable environmental conditions [53]. The plant having more scavenging enzymes and osmoprotectants can resist more to unfavorable conditions [9,14], specifically under water-deficit [8,10]. Our results showed that, VM4 produced more scavenging enzymes and osmoprotectants than VM2 in leaves and roots under both water-deficit regimes (Figs 2 and 3). Interestingly PRO contents were higher in the leaves of VM2 as compared to VM4 under slow water-deficit. This indicates that VM4 cope t water-deficit stress with PRO content more efficiently in roots as compared to leaves. The AC and TPC increased in leaves and roots of both rootstocks under water-deficit regimes. Plants increased the accumulation of TPC by activating biosynthesis pathways which and inhibited oxidation [54]. Tolerant rootstocks showed more AC and TPC than sensitive [8].

Potassium is major component of photosynthetic machinery that helps in opening and closing of stomata. When plants are exposed to water-deficit, potassium concentration significantly decreased, resulting in the closure of stomata and oxidative damage. Leaves of VM4 showed no significant change in potassium content under tested water-deficit regimes, while VM2 recorded a decrease in leaves potassium content suggesting that roots of VM4 transported of potassium ions to leaves in order to favor photosynthetic machinery as compared to VM2. Similar findings were also observed by García-Sánchez et al. [55] showing decrease in potassium content in roots of sensitive wheat genotypes under water-deficit condition. The calcium concentration was slightly increased in the leaves and roots of VM4 and VM2 under water deficit condition (Figs 4 and 5). The nitrogen and phosphorous were significantly decreased in leaves and roots of both rootstocks. Nitrogen concentration, its uptake and assimilation were decreased due to abundance of nitrogen dilution [56]. Nitrogen and phosphorous uptake from soil are decreased under low soil moisture [57,58]. The sodium and chloride concentrations were not affected by water-deficit. However, VM4 roots showed slight increase in chloride concentration under slow water-deficit (Fig 5).

The article "Physiological and biochemical responses of Kinnow mandarin grafted on diploid and tetraploid Volkamer lemon rootstocks under different water-deficit regimes" was retracted in 2022. Reasons: compromised peer review; a conflict of interest; concerns about the authorship.

In conclusion, both rootstock-scion combinations recorded noticeable changes in metabolic processes under tested water-deficit regimes (Fig 8). As, 2x and 4x plants presented differences in their anatomical, physiological processes and tolerance mechanism, they also showed difference in the induction of tolerance mechanism against water scarcity when grafted with KM (Fig 8). The VM4 showed more tolerance by maintaining photosynthetic machinery, strong antioxidant defense mechanism, better conductivity and uptake of plant nutrients. The VM4 plants showed less decrease in *Pn*, *gs*, *E*, Fv/Fm, Fv´/Fm´, LSA and RWC and less increase in NPQ as compared to VM2 indicating its tolerance against water-deficit (Fig 8). The SOD, POD, CAT, APx, GR, PRO and GB were also higher in VM4 thanVM2 under water-deficit. Tested rootstock-scion combinations exhibited early response to fast water-deficit as compared to slow water-deficit. Both rootstock-scion combinations quickly responded to water deficit; however, response of VM4 to cope the adverse effect of stress was more efficient than VM2. Moreover, both rootstock-scion combinations showed slow and adaptive response, while VM4 showed quick adaptive response because of better antioxidant defense mechanism. In the field, there is yet very limited information about the behavior of this innovative plant material. Such investigations should be performed in the field. Further studies required to observe the fruit characteristics of both genotypes and their phytochemical compounds [59].

**Fig 8:** Schematic diagram of physiological and biochemical responses of VM4 and VM2 under fast and slow water-deficit conditions.

The article "Physiological and biochemical responses of Kinnow mandarin grafted on diploid and tetraploid Volkamer lemon rootstocks under different water-deficit regimes" was retracted in 2022. Reasons: compromised peer review; a conflict of interest; concerns about the authorship.

## Supporting information

S1 Fig Measurements of the leaf morphological parameters under different water-deficit regimes. (A, B) relative water content; (C, D) leaf surface area in the leaves of VM4 and VM2. Values are mean ± S.E. at p < 0.05 (n = 3). ⚫ = VM4 control; ○ = VM4 water deficit; ▼ = VM2 control; Δ = VM2 water deficit.
(DOCX)

S2 Fig Measurements of the oxidative markers and biochemical compounds in the leaves of VM4 and VM2 grown under fast and slow water-deficit regimes. (A) hydrogen peroxide; (B) malondialdehyde; (C) antioxidant capacity; (D) total phenolic content; (E) shoot dry biomass; (F) root dry biomass. ⬛ = VM4; ⬜ = VM2. Values are mean ± S.E. at p < 0.05 (n = 3).
(DOCX)

S3 Fig Measurements of the oxidative markers and biochemical compounds in the roots of VM4 and VM2 grown under fast and slow water-deficit regimes. (A) hydrogen peroxide; (B) malondialdehyde; (C) antioxidant capacity; (D) total phenolic content; (E) shoot dry biomass; (F) root dry biomass. ⬛ = VM4; ⬜ = VM2. Values are mean ± S.E. at p < 0.05 (n = 3).
(DOCX)

S1 Table Mean values of VM4 and VM2 under slow and fast water deficit regimes. (DOCX)

S2 Table Analysis of variance of VM4 and VM2 under slow and fast water deficit regimes. (DOCX)
